# A Case Study of Multiple Maintenance Efficacy in Gynaecological Surgery Assessed by Deep Learning

**DOI:** 10.1155/2022/8574000

**Published:** 2022-08-08

**Authors:** Yanmei Zheng, Qi Yuan

**Affiliations:** ^1^Department of Operating Room Nursing, West China Second University Hospital, Sichuan University/West China School of Nursing, Sichuan University, Chengdu, Sichuan 610000, China; ^2^Key Laboratory of Birth Defects and Related Diseases of Women and Children, Ministry of Education, Sichuan University, Chengdu, Sichuan 610000, China

## Abstract

Deep learning is a new learning concept and a highly effective way of learning, which is still being explored in the field of nursing education. This paper analyses the effectiveness of interventions in perioperative gynaecological care using humanised care in the operating theatre and the impact of this model of care on patients' psychological well-being and sleep quality. A deep learning-based vision robot was designed to provide higher quality of care for our human care and simplify our approach to gynaecological surgery. The anxiety and depression scores of the two groups were significantly improved after and before care, and the scores of the observation group were lower than those of the control group, with a statistically significant difference (*P* < 0.05). The humanised care for gynaecological surgery patients in the perioperative period is more conducive to the improvement of their negative emotions and at the same time can improve the sleep quality of patients, so it can be further promoted.

## 1. Introduction

As a source of stress, gynaecological surgery does not reduce the psychological disturbance and adverse effects on patients, which requires nursing interventions in parallel with the surgery, in the hope of improving the psychological state of patients and their sleep quality [1].

Humanised care is a model of care based on conventional care, which pays more attention to the physical and mental health of the patient, formulating a care plan that is tailored to each patient's specific physical and mental state, and which also shows respect for the differences in gynaecological surgery patients [2].

In addition, the use of humanised care in gynaecological surgery has brought patients and nurses closer together and provided an important guarantee of safety in the operating theatre, which has positive implications for the health and long-term development of the doctor-patient relationship [3]. The results of this study suggest that the anxiety and depression of the patients who received humanised care in the operating theatre improved significantly, suggesting that this model of care is conducive to improving the psychological well-being of the patients. At the same time, patients with humanised care services in the operating theatre slept longer after surgery, which indicates that this model of care has a positive impact on prolonging patients' sleep time and improving sleep quality and that the improved sleep quality of patients also ensures the nutrition supply of the body to a large extent, which is also important for postoperative recovery [4].

Operating theatre nursing is characterised by high workload, long working hours, high technical requirements, and high risks, especially in gynaecological operating theatres [5]. Therefore, for gynaecological surgery patients, it is important to strengthen clinical perioperative nursing interventions for patients. Humanised care reflects respect for individual differences, and this model of care is therefore recognised and supported by the majority of patients [6].

With the addition of vision, the robot is able to observe the external environment, process the information from the camera, and obtain information about the object to be grasped based on the information from the camera [7]. Similarly, vision robots are able to locate objects, and with the combination of object recognition and vision positioning, the exact coordinates of the object to be grasped can be obtained. The advent of artificial intelligence has not only brought about ideas but also many technological changes that are leading the way in vision robots [8]. Deep learning has not only allowed vision robots to shed their bulky shells but has also made them smarter than ever, and some have even developed ideas and minds of their own. Artificial intelligence has also become a technology hit now and is now being used in a variety of fields, changing traditional production processes and habits. The artificial intelligence robotics industry is now driving business growth [9].

Faced with the negative impact of informing nursing, the use of an in-depth learning approach in gynaecological nursing guides gynaecological patients in evaluating evidence of practice and encourages gynaecological patients to engage in self-directed learning, thereby developing nurses' metacognitive skills and critical thinking. This paper examines the use of an in-depth learning model in clinical nursing to train nurses in emergency clinical skills [10].

## 2. Related Work

The results of the survey indicate that nursing students have some awareness of deep learning but are at a low to moderate level and need to be improved. A number of studies have shown that the educational environment is positively correlated with the level of deep learning and that a good educational support environment is an important prerequisite for the creation of a learning environment and access to learning resources [11]. A semistructured interview to explore nurses' perceptions of the teaching and learning environment showed that effective classroom teaching and learning environment is a catalyst for nurses' use of deeper learning [12]. The survey identified that medical students generally adopted three learning styles, in-depth learning, surface learning, and strategic learning, and that they were able to adapt their learning methods to the changing teaching environment in a timely manner. [13] pointed out that nurses' sense of self-efficacy in online learning is an important influence on deep learning, and that a good sense of self-efficacy among nurses can positively predict and guide the development of deep learning, and that level of education, network skills, and self-directed learning also have an impact on the level of deep learning. However, some studies suggest that there is disagreement about the impact of general demographic characteristics such as gender, grade, and profession on the production of deeper learning styles, and further research is needed [14, 15].

The study reported that the use of clinical nursing experience alone is not effective in facilitating the development of advanced learning and that only trainee nurses engaged in advanced learning can take the initiative to develop the creative and participatory skills to master the whole-patient model of care [16, 17]. Lectures on human anatomy and physiology are based on an in-depth learning pathway that takes full advantage of the learning community to teach students to solve complex problems to complete the transfer of knowledge. In [18], an online postclinical pilot study was conducted in which nurse educators guided students through a complex clinical environment. Students were able to structure conversations in a face-to-face or online environment to successfully deal with complex or acute clinical patients, developing their integrative skills such as clinical scenarios and guided discussions.

## 3. Binocular Vision System for Nursing Robots

### 3.1. The Overall Process of the Care Robot

The main work of this paper is to build a set of deep learning-based vision servo system for nursing robots; the main function of the system is to complete some basic actions of the home robot and to autonomously complete the tasks assigned to it by the master, for example, a simple operation like grasping a cup; the master just needs to issue a voice command to grasp the cup, and the nursing robot can autonomously find the cup in the field of view and can autonomously grab the cup. To design such a care robot, it is important to have an overview of the whole system, to understand the types of signals and the sequence of the various stages [19]. As voice control is used, there must be recognition of speech. There is the grasping of the cup, so there is the creation of a three-dimensional coordinate system for vision, as well as object recognition. All these technologies are key to researching nursing robots today.

The main purpose of designing this care robot is to play a role in caring for people who are inconvenienced and to help them with the daily operations of life. The workflow of the care robot for grasping objects in a practical application is described here, as shown in Figure 1.

As shown in Figure 1, the main steps in its mode of operation are as follows.

In the first step, the care robot acquires an external voice signal, which is a specific human voice signal, not only for convenience but also to prevent interference from other people's voices and for greater security.

In the second step, the PC processes the voice signal, analyses the voice commands, and makes the care robot act accordingly, which is much faster.

The third step is to accept the acquired voice commands, capture the image with the binocular camera, find the target object in the image, and obtain the coordinates of the object.

In the fourth step, a neural network is used to correct the coordinate information of the target and then perform the grasping action.

### 3.2. Human-Specific Speech Recognition for Care Robots

The original intention of the deep learning-based care robot design was to have artificial intelligence, so to be as flexible and the control signals as simple as possible, and after comparing other control signals, the one chosen was the voice signal. There are three main advantages.

Firstly, the use of a voice signal also ensures that the person giving the command only needs to wear a wireless headset and send voice commands within a certain range. Traditional command outputs often require the user to be right next to the machine, and the use of voice input solves this problem.

Secondly, the functions that can be added by using voice signals are often more than those of hardware input, and it is not necessary to consider the number of voice commands, but traditional hardware is different; after all, more signals require more hardware to distinguish the type of signal, using voice input solves this problem and is also more convenient for us to control.

Thirdly, the choice of specific human voice recognition can also play a major role in preventing interference from other people's voices and can increase the stability of the input signal.

The advantage of choosing a headset plus a computer processing method is mainly to determine the distance between the sound source and the receiver, which can effectively control the decibel level of the sound, thus allowing better recognition and reducing recognition errors. As this experimental platform uses a one-to-one service, the recognition of the voice signal must be person specific so as to ensure that the care robot has as little influence on the outside world as possible [20].

The main method used to acquire the speech signal is the recognition of isolated words for person-specific speech recognition. The training of the person-specific speech is carried out, and the specific process includes the following steps.

**Step 1 .**

The acquired person-specific speech signal sequence *X*(*n*) is preprocessed to obtain a new speech sequence Youm(*n*) after which a Fourier transform is applied to it:

(1) $$\begin{array}{c} X\left(i,k\right)=\text{FFT}\left[X_{\text{m}}\left(n\right)\right]. \end{array}$$

Universal line energy:

(2) $$\begin{array}{c} E\left(i,k\right)={\left[X\left(i,k\right)\right]}^{2}. \end{array}$$

**Step 2 .**

Filtered by *H*_*m*_(*k*) filter phantom,

(3) $$\begin{array}{c} H_{m}\left(k\right)=\left\{\begin{array}{cc} \frac{k-f\left(m-1\right)}{f\left(m\right)-f\left(m-1\right)}, & f\left(m-1\right)\leq k\leq f\left(m\right),\\ \frac{f\left(m+1\right)-k}{f\left(m+1\right)-f\left(m\right)}, & f\left(m\right)\leq k\leq f\left(m+1\right),\\ 0,0\leq k\leq f\left(m-1\right), & f\left(m+1\right)<k. \end{array}\right. \end{array}$$

In equation (3), 0 ≤ *m* ≤ *M*, *M* is the number of filters *H*_*m*_(*k*).

Energy after *H*_*m*_(*k*) filter:

(4) $$\begin{array}{c} S\left(i,k\right)=\overset{N-1}{\underset{k=0}{\sum }}E\left(i,k\right)H_{m}\left(k\right),0\leq m\leq M. \end{array}$$

**Step 3 .**

Calculate the characteristic parameters of MFCC:

(5) $$\begin{array}{c} \text{mfcc}\left(i,n\right)=\sqrt{\frac{2}{M}}\overset{M-1}{\underset{m}{\sum }}\log\left[S\left(i,m\right)\right]\cos\left(\frac{\pi n\left(2m-1\right)}{2M}\right). \end{array}$$

**Step 4 .**

The feature matrix calculated is saved with the command in the form of a file name, which is matched when a speech signal is received to determine the speech command and obtain the object to be grasped.

The main idea of using the DTW algorithm is to use the global minimum method, comparing the template calculated by the DTW algorithm with the implementation of the saved template, if the shortest distance from one of the templates, the corresponding content is the command of that saved template.

### 3.3. Vision Coordinate System Establishment for the Nursing Robot

After the care robot receives the voice signal, the computer matches the corresponding command, and then, it enters the vision part, which needs to make corresponding actions to the voice signal, identify the object to be grasped, and grasp the object to be grasped and needs to get the 3D coordinates of the grasped object, where the 3D coordinates are obtained by establishing a binocular vision coordinate system, modelling the visual space to facilitate the later identification and grasping action of the robot arm.

The images captured using a single camera are two-dimensional and lack depth information. The addition of a camera is also used to calculate the depth information by comparing the difference in coordinates of the same point in two images through a parallax map. (Based on observations and experiments, it was found that the *X* coordinate of the object in the right view is different from the left view, but the *F* coordinate is the same, and the parallax is set to *Z*.) The coordinates of point *P* in the left and right camera are different, but in practice, it is just a point, and the coordinates of this point are set to *p*(*x*, *y*, *z*). The following conclusions can be drawn from the triangulation.

(6) $$\begin{array}{c} A\left(x,\right)=f\frac{x}{z}, \end{array}$$

(7) $$\begin{array}{c} B\left(x,\right)=f\left(\frac{x-d}{z}\right), \end{array}$$

(8) $$\begin{array}{c} A\left(,\text{y}\right)=B\left(,y\right)=f\frac{y}{z}, \end{array}$$

(9) $$\begin{array}{c} D=A\left(x,\right)-B\left(x,\right). \end{array}$$

After calculation, we get

(10) $$\begin{array}{c} x=\frac{B\cdot A\left(x,\right)}{D}, \end{array}$$

(11) $$\begin{array}{c} y=\frac{B\cdot A\left(,y\right)}{D}=\frac{B\cdot B\left(,y\right)}{D}, \end{array}$$

(12) $$\begin{array}{c} Z=\frac{B\cdot f}{D}. \end{array}$$

The coordinates of the object calculated by the above formula are the coordinates under the camera; if you want to get the image coordinates, you need to do the following process.

As shown in Figure 2, the process of establishing a 3D coordinate system with the binocular camera is actually the process of transforming the coordinate system to obtain the real coordinates of the object in reality. After establishing the 3D coordinates, the experimental verification was carried out on the same platform as the voice platform, both being MFC projects under Windows.

## 4. Case Studies

### 4.1. General Information

From October 2019 to June 2020, 200 patients who underwent gynaecological surgery in the operating room of our hospital were selected as the subjects of the study and were divided into a control group and an observation group according to the random number table method, with 100 patients in each group. The average age of the control group was 22-68 years, 46.26 ± 1.82 years old; the average age of the observation group was 23-69 years old, 46.29 ± 1.87 years old. The general data of the two groups were not statistically significant (*P* > 0.05) and were comparable. The study was approved by the ethics committee of the hospital, and the patients gave their informed consent.

### 4.2. Results

The negative emotions of both groups improved after care, and the negative psychological scores of patients in the observation group were significantly lower than those in the control group after care, with statistically significant differences (*P* < 0.05) (see Table 1).

The sleep time of the two groups was counted at 1 d, 3 d, and 7 d postoperatively, and the results showed that the sleep interval of the observation group was significantly longer than that of the control group at each time point (see Table 2).

As can be seen from Figure 3, the function fitness value reaches its optimal value after almost 35 iterations, and in subsequent iterations, the function fitness value does not fluctuate or jump massively and basically tends to be stable. The genetic algorithm optimises the BP neural network to a certain extent to avoid the difficulties of tuning the parameters and on the other hand to find better parameters more quickly.

The application of CNN to a nursing robot not only solves the problem of object recognition when the robot arm grasps an object but also allows this to be combined with the grasping state of the robot arm. The role of object recognition in a nursing robot is not only to mark the object but also to give the robot arm advice on how to grasp the object by recognising it. This increases the gripping stability of the nursing robot, as shown in Figure 4.

## 5. Conclusion

This paper describes the overall structure of the deep learning-based nursing robot vision system and provides an in-depth study of the control strategy of the deep learning-based nursing robot vision system. The human-specific speech recognition part of the nursing robot was completed, mainly using the DTW algorithm, and experimental validation was carried out to demonstrate the accuracy of the DTW algorithm used on speech-isolated word signals. The theoretical derivation of the 3D coordinate system established by the binocular camera and the elaboration of the specific operation steps were carried out, and the upper computer was programmed to experimentally verify the application of the 3D coordinate system established by the binocular vision in the nursing robot.

## Figures and Tables

**Figure 1:** Flow of a care robot grasping an object.

**Figure 2:** Coordinate transformation.

**Figure 3:** Deep learning training and care outcomes.

**Figure 4:** Nursing robot gripping effect.

**Table 1:** Intergroup comparison of pre- and postcare adverse psychological scores ($\bar{x}\pm s$, scores).

Group	Anxiety score	Depression score
Observation group (*n* = 100)		
Before nursing	15.23 ± 2.26	16.89 ± 2.33
After nursing	7.41 ± 0.15	7.32 ± 0.52
Control group (*n* = 100)		
Before nursing	15.43 ± 2.28	16.78 ± 2.54
After nursing	12.42 ± 0.22	12.49 ± 0.48

**Table 2:** Comparison of sleep duration between groups ($\bar{x}\pm s$, h).

Group	One day after operation	Three days after operation	Seven days after operation
Observation group (*n* = 100)	6.88 ± 0.12	7.49 ± 0.56	8.11 ± 0.27
Control group (*n* = 100)	5.23 ± 0.26	5.85 ± 0.22	6.01 ± 0.22
*T* value	57.621	27.256	60.295
*P* value	0	0	0

## Data Availability

The dataset used in this paper are available from the corresponding author upon request.
